# The Association between the rs312457 Genotype of the SLC16a13 Gene and Diabetes Mellitus in a Chinese Population

**DOI:** 10.1155/2021/9918055

**Published:** 2021-06-26

**Authors:** Hui Zheng, Suying Pu, Yu Zhang, Yujuan Fan, Jialin Yang

**Affiliations:** ^1^Department of Endocrinology and Metabolism, Minhang Hospital, Fudan University, 170 Xin-Song Road, Shanghai 201199, China; ^2^Department of Neurology, Shanghai Xuhui District Dahua Hospital, 909 LaoHuMin Road, Shanghai 200237, China

## Abstract

**Objective:**

SLC16a genes encode H + -coupled monocarboxylate transporters (MCTs). MCTs are involved in maintaining interstitial fluids' pH and regulating insulin's binding affinity to its receptor, which is a potential mechanism for the onset of diabetes. In this research, we make explorations of the association between the rs312457 genotype of the SLC16a13 gene and diabetes in the Chinese population.

**Methods:**

It included 384 type 2 diabetes patients and 1,468 healthy control subjects in total. We measured the anthropometric parameters, glycaemic index, homeostasis model assessment-B cell (HOMA-%B), lipid profile, and homeostasis model assessment-insulin resistance (HOMA-IR). The associations between the rs312457 genotype and type 2 diabetes were analyzed.

**Results:**

The rs312457 genotype was markedly in relation to type 2 diabetes (*P* = 0.002). The frequency of the rs312457 risk allele (G) was 4.8%, higher than that of the wild-type allele (A) in patients of type 2 diabetes, indicating that allele (G)'s presence seemed to make the risk of type 2 diabetes go up. Compared to the GA and AA genotypes, the GG genotype of rs312457 significantly increased the risk of contracting diabetes mellitus (*P* ≤ 0.001). Moreover, the rs312457 genotype was associated with HOMA-%B. Subjects harbored the GG genotype of rs312457, whose HOMA-%B level went down in comparison with that in subjects harboring the AA genotype (*P* = 0.023).

**Conclusion:**

Our results revealed that the rs312457 genotype of the SLC16a13 gene was correlated with the development of diabetes mellitus in the Chinese population.

## 1. Introduction

As a complicated metabolic disease, diabetes mellitus is a characteristic of elevated blood glucose due to insulin secretion and/or deficiency. Long-term poor glycaemic control of diabetic patients can be accompanied by a variety of complications and organ dysfunction or failure, especially in the eyes, heart, blood vessels, kidney, and nervous system. Diabetes has gradually become a focus of public health worldwide, and China ranks first in the number of diabetic patients worldwide. In 2013, it was reported by Ning et al. [1] that as for Chinese adults, the overall incidence of diabetes was estimated to be 11.6%, with rates of 12.1% for males and 11% for females. Recently, the incidence of diabetes is estimated to be 8.1%. Diabetes is a serious health problem and a heavy burden in China.

There is an urgent need for strategies for preventing and treating diabetes to control the spread of the disease. Type 2 diabetes (T2D) results from *β*-cell dysfunction and/or insulin resistance, which is facilitated due to multifactorial genetic factors [2]. In examining the genetic mechanism of diabetes mellitus, candidate gene approaches, linkage analysis, genome-wide association studies (GWAS), and large-scale association studies have managed to recognize numerous loci which contribute to T2D susceptibility [3–6]. The research of gene polymorphism is becoming more and more popular, which helps to discover new genes related to T2DM susceptibility [7]. Related reports indicate that the rs4430796 single nucleotide polymorphism (SNP) of HNF1*β* gene is associated with type 2 diabetes in the elderly [8]. In gestational diabetes, a significant difference was found between grade B and D diabetes of CC and TC genotypes of rs2975760 and grade B and D diabetes of TT genotypes. Compared with the GG genotype, the B and D diabetes of the AA and AG genotypes of rs3792267 are significantly different, and the allele A is significantly increased than the allele G. In 2014, Hara et al. identified three novel loci for T2D by GWAS, one of which was the rs312457 loci of the SLC16a13 gene [9]. The SLC16a gene encodes H + -coupled monocarboxylic acid transporters (MCTs) [10]. MCTs are involved in maintaining the pH of the interstitial fluid and regulating the binding affinity of insulin to its receptor [11], which is a potential mechanism for the onset of diabetes. However, the role of the rs312457 locus of the SLC16a13 gene in the pathogenesis of diabetes has not been reported yet. To determine whether the genetic variations of SLC16a13 are associated with T2D in Chinese patients, we also selected rs312457 as a single nucleotide polymorphism (SNP) tag in the SLC16a13 gene and analyzed its relation to T2D.

## 2. Methods and Materials

### 2.1. Study Subjects

1,852 subjects, including a total of 1,468 nondiabetic controls and 384 patients with T2D, were recruited from Minhang Hospital, Fudan University in Shanghai. The following inclusion criteria were utilized for the controls: (1) fasting plasma glucose (FPG) < 6.1 mmol/L and (2) postprandial plasma glucose (PPG) < 7.8 mmol/L. Since 1999, T2DM has been diagnosed by the World Health Organization (WHO) as having the following characteristics: FPG ≥ 7.0 mmol/L and/or 2 hours postprandial plasma glucose ≥ 11.1 mmol/L. In this group, diabetes was diagnosed no more than 6 months ago, and the subjects did not receive insulin therapy. All participants were Chinese Han individuals who lived in Shanghai. The Ethics Committee of the Minhang Hospital, Fudan University approved this research and it was implemented in conformity to all ethical guidelines. We gained written informed consent for an interview and a blood sample donation from each participant.

### 2.2. Anthropometric and Clinical Measurements

We collected anthropometrical measurements of weight, blood pressure, height, and the waist-to-hip ratio (WHR). We calculated BMI as weight (in kg) divided by height (in m^2^). We collected plasma samples after a 12-hour overnight fast. We measured the FPG, low-density lipoprotein cholesterol (LDL-C), high-density lipoprotein cholesterol (HDL-C), total cholesterol (TC), and triglycerides (TG) levels by making use of standardized enzymatic procedures (Hitachi 7600-110 automatic biochemical analyzer; Hitachi Ltd, Tokyo, Japan). We detected C peptide and plasma insulin (INS) by making use of radioimmunoassay. Glycosylated haemoglobin (HbA1C) was detected by making use of an HLC-723G7 TOSOH analyzer (TOSOH Ltd, Tokyo, Japan).

### 2.3. The Selection of Single Nucleotide Polymorphism (SNP) and Genotyping

rs312457 was selected based on previous reports from Japan. The detection of rs312457 was performed by the Shanghai OEbiotech Company using Sequenom MassARRAY SNP technology [12]. The genotyping success rate was 99.74%. The frequencies of the genotypes conformed to Hardy-Weinberg equilibrium (HWE) (*P* > 0.05).

### 2.4. Deoxyribonucleic Acid (DNA) Extraction

Extracted from the whole blood genome, DNA was analyzed by making use of 1% agarose gel electrophoresis, and we subsequently estimated the concentration and DNA degradation degree. We applied quality inspection aiming at gaining the DNA A260/A280 ratio (OD) which was in the range of 1.8 to 2.0, with a DNA concentration of more than 50 ng/*μ*L and good quality gel electrophoresis bands. DNA was then transferred to 96-well plates and stored at -20°C for further analysis.

### 2.5. Statistical Analysis

PLINK 1.9 was used to explore the relationship between rs312457 and T2D. The results were expressed in the form of the means ± standard deviation (SD) or as a ratio. The comparison of alleles and genotype distribution in the T2D and controls was performed using *χ*^2^ tests. We compared quantitative traits among different genotypes by making use of analysis of variance (ANOVA). The HWE in the control subjects was analyzed by PLINK 1.9. We performed power calculations by making use of Quanto v1.2.4. We performed other statistical analyses by making use of SPSS (version 19.0; SPSS Institute Inc.). We considered a *P* value less than 0.05 significant from the perspective of statistics.

## 3. Results

### 3.1. Study Characteristics of Populations

We showed the anthropometric and biochemical features of the study subjects in Table 1. SNP genotyping (RBMS1–RS 7593730 and BCAR1-RS 7202877) was performed on 991 T2DM patients and 970 nondiabetic controls, and their correlation with T2DM was analyzed. The gender distribution (*P* = 0.191) and LDL-C distribution (*P* = 0.787) between the case and control group were not statistically different. The two groups were obviously different with respect to HbA1C, FBG, HOMA-%B, and HOMA-IR values (*P* < 0.05). The groups did not obviously differ in other characteristics.

### 3.2. Characteristics of rs312457

We presented the features of rs312457 (including its genotype frequency, position and minor allele frequency, and MAF) in Table 2. rs312457 was located at chr17 : 7037074, which was an intron variant on SLC16A13. The alleles of rs312457 were G/A. Compared with the control group, the MAF of the T2D group increased significantly. All genotypes were distributed in conformity to HWE.

### 3.3. Allele Frequencies of rs312457 and Genotype Distribution

We presented the allele frequencies of rs312457 in Table 3. Carriers of the rs312457 risk allele (G) had a 4.8% increased risk of T2D in comparison with carriers of the wild-type allele (A) (*P* ≤ 0.001, OR 1.25, 95% CI 1.06-1.48); therefore, the presence of the G allele seemed to make the risk of T2D go up. The genotype distribution was shown in Table 4. The GG genotype of rs312457 was in relation to increased diabetes risk (*P* < 0.05).

### 3.4. Relationships between rs312457 and Quantitative Traits

The HOMA-%B of subjects carrying the GG genotype obviously fell off in comparison with that of subjects with the AA genotype (*P* < 0.05), and GG carriers had increased HbA1C levels (*P* < 0.05). None of the polymorphisms exhibited a significant correlation with the BMI, WHR, and blood lipid levels in diabetes patients (Table 5).

## 4. Discussion

Fourteen SLC16a genes that encode the monocarboxylate transporters (MCTs), including MCT1-MCT14, have been identified [13, 14]. The structures of all MCTs include a large intracellular loop, intracellular N- and C- termini, and 12 transmembrane domains (TMDs) [15]. Among family members, the greatest variation is exhibited through making use of the N- and C-termini and the large loop between TMDs 6 and 7, whereas the TMDs are highly retained. MCT1-4 transports single carboxylic acid molecules, such as lactic acid, pyruvic acid, and ketones [16]. MCT8 mainly transports thyroid hormones, including T3 and T4 [17, 18]. MCT10 participates in the bidirectional transport of iodothyronines and aromatic amino acids [19, 20]. MCT10 tends to transport MCT8 even less effectively than T3 [21]. The SNPs in the SLC16a gene can change the protein sequence of MCTs, which may lead to differences in tissue distribution and function. However, the regulatory mechanism of the change in the protein sequence of MCTs caused by the SLC16a gene in diabetes was still unclear.

MCTs are H + -coupled [22] and involved in the maintenance of the pH of interstitial fluids [11]. Interstitial fluids allow extracellular signalling molecules, such as neurotransmitters and hormones, to achieve the regulation of cell function. Interstitial fluid's pH alteration influences the efficiency of intracellular signalling transduction by extracellular signalling molecules, including insulin. In skeletal muscle, reduced extracellular pH values of interstitial fluid reduce insulin's binding affinity to its receptor, which is in relation to a reduction of insulin receptor phosphorylation (activation) while the expression of the insulin receptor on the plasma membrane of skeletal muscle has no changes [23]. Thus, MCTs participated in insulin resistance by reducing insulin's binding affinity to its receptor.

In our study, the rs312457 genetic variation in SLC16a13 increased the risk of diabetes. Subjects carrying the GG genotype of rs312457 had the highest risk of diabetes. As for subjects who carried the GG genotype of rs312457, basal insulin secretion, as evaluated by HOMA-%B, was reduced. That finding suggested that rs312457's genetic variations in SLC16a13 might be in relation to pancreatic insulin secretion. We did not identify a relationship between rs312457 and HOAM-IR in diabetic patients. This result might suggest that pancreatic secretion of diabetes patients decreased faster with insulin resistance in individuals who carried the homozygous GG genotype of rs312457. Given that MCTs exhibited tissue distribution specificity, the functions of MCTs in various tissues differed. Therefore, MCTs may also participate in regulating pancreatic *β*-cell function in the pancreas of diabetic patients.

We need to put further efforts into identifying the mechanism of SLC16a13 in the pathogenesis of diabetes mellitus and facilitate strategies of early diagnosis and preventative aiming at reducing this increased disease burden. As a kind of emerging discipline, pharmacogenomics emphasizes the function of genetic variations which are inherited and acquired, in drug responses as well as facilitates appropriate selection of antidiabetic drugs.

To the best of our knowledge, this study confirmed for the first time that the rs312457 genotype of the SLC16a13 gene was associated with diabetes in the Chinese population. This study provides new and useful information for the study of the underlying mechanism of diabetic patients and helps the appropriate choice of antidiabetic drugs.

However, this study has limitations. Since the control was recruited from the hospital, a certain degree of selection bias cannot be ruled out. However, in the current sample, the population is relatively homogeneous. The subjects all live in the same area and have the same dietary preferences in terms of the ratio of fat to carbohydrate. Under current conditions, the potential selection bias is considered to be the smallest.

## Figures and Tables

**Table 1:** Comparing clinical and biochemical features between the two groups.

	Controls	T2DM	*P*
	*n* = 1468	*n* = 384	
Age (years)	58.87 ± 14.06	59.58 ± 15.83	0.397
Sex (male/female)	824/644	219/165	0.751
BMI (kg/m^2^)	24.89 ± 3.80	25.28 ± 4.05	0.109
WHR	0.93 ± 0.06	0.94 ± 0.06	0.060
Systolic BP (mmHg)	127.47 ± 14.10	128.03 ± 14.79	0.493
Diastolic BP (mmHg)	79.16 ± 7.71	79.23 ± 7.90	0.871
FBG (mmol/L)	5.01 ± 0.63	9.03 ± 3.56	0.001^∗^
HbA1C (%)	5.49 ± 0.23	10.41 ± 2.71	0.001^∗^
TC (mmol/L)	4.46 ± 1.20	4.58 ± 1.40	0.086
TG (mmol/L)	2.09 ± 2.57	2.19 ± 2.98	0.495
HLD-C (mmol/L)	1.00 ± 0.37	1.01 ± 0.40	0.670
LDL-C (mmol/L)	2.64 ± 0.90	2.70 ± 1.00	0.228
HOMA-%B	78.59 ± 49.91	44.92 ± 28.78	0.001^∗^
HOMA-IR	1.49 ± 0.97	1.75 ± 1.11	0.001^∗^

Data are presented as the means ± standard deviation or as ratios. ^∗^*P* value < 0.05.

**Table 2:** Main features of rs312457.

SNP	Chromosome	Position	Alleles (risk/other)	MAF		*P*
				Controls	T2DM	
rs312457	17 : 7037074	Intron	G/A	0.12	0.17	0.002^∗^

^∗^ *P* value < 0.05.

**Table 3:** Allele frequencies of rs312457.

SNP	Controls (%)		T2DM (%)		*P* value	OR (95% CI)
	G	A	G	A		
rs312457	343 (12.3)	2,457 (87.8)	131 (17.1)	637 (82.9)	0.001^∗^	1.25 (1.06-1.48)

^∗^ *P* value < 0.05.

**Table 4:** Genotype distribution of the rs312457 polymorphism in control subjects and T2DM patients.

SNP	Controls (%)			T2DM (%)			*P*
	GG	GA	AA	GG	GA	AA	
rs312457	16 (9.8)	99 (43.4)	269 (46.8)	16 (23.1)	311 (27.1)	1073 (49.8)	0.001^∗^

^∗^ *P* value < 0.05.

**Table 5:** Comparison of mensurable traits among rs312457 variants.

	rs312457			*F*	*P*
	GG	GA	AA		
BMI (kg/m^2^)	26.24 ± 6.46	25.40 ± 3.95	25.17 ± 3.91	0.507	0.603
WHR	0.96 ± 0.09	0.94 ± 0.07	0.93 ± 0.06	1.658	0.192
HbA1C (%)	12.12 ± 2.42	10.39 ± 2.70	10.38 ± 2.61	3.353	0.036^∗^
HOMA-%B	33.78 ± 25.52	39.50 ± 26.48	47.56 ± 29.42	3.799	0.023^∗^
HOMA-IR	1.62 ± 1.07	1.66 ± 0.92	1.78 ± 1.12	0.497	0.609
TC (mmol/L)	4.42 ± 1.02	4.54 ± 1.13	4.61 ± 1.50	0.186	0.830
TG (mmol/L)	1.80 ± 1.42	2.35 ± 3.01	2.16 ± 3.05	0.278	0.757
HDL-C (mmol/L)	0.97 ± 0.24	1.02 ± 0.30	1.01 ± 0.43	0.098	0.907
LDL-C (mmol/L)	2.63 ± 0.99	2.64 ± 0.87	2.73 ± 1.04	0.345	0.708

^∗^ *P* value < 0.05.

## Data Availability

The datasets used and/or analyzed during the current study are available from the corresponding author on reasonable request.
